This article has been retracted.

# MiR-203 Suppresses ZNF217 Upregulation in Colorectal Cancer and Its Oncogenicity

**DOI:** 10.1371/journal.pone.0116170

**Published:** 2015-01-26

**Authors:** Zewu Li, Lutao Du, Zhaogang Dong, Yongmei Yang, Xin Zhang, Lili Wang, Juan Li, Guixi Zheng, Ailin Qu, Chuanxin Wang

**Affiliations:** Department of Clinical Laboratory, Qilu Hospital, Shandong University, Jinan, Shandong Province, China; The University of Hong Kong, CHINA

## Abstract

Zinc finger protein 217 (ZNF217) is essential for cell proliferation and has been implicated in tumorigenesis. However, its expression and exact roles in colorectal cancer (CRC) remain unclear. In this study, we demonstrated that ZNF217 expression was aberrantly upregulated in CRC tissues and associated with poor overall survival of CRC patients. In addition, we found that ZNF217 was a putative target of microRNA (miR)-203 using bioinformatics analysis and confirmed that using luciferase reporter assay. Moreover, in vitro knockdown of ZNF217 or enforced expression of miR-203 attenuated CRC cell proliferation, invasion and migration. Furthermore, combined treatment of ZNF217 siRNA and miR-203 exhibited synergistic inhibitory effects. Taken together, our results provide new evidences that ZNF217 has an oncogenic role in CRC and is regulated by miR-203, and open up the possibility of ZNF217- and miR-203-targeted therapy for CRC.

## Introduction

Colorectal cancer (CRC) is the second and third most common malignant tumor in females and males, respectively, worldwide, with over 1.2 million new cases and an estimated 608,700 deaths in 2008 alone [1]. Despite recent advances in the diagnosis and treatment of CRC, the overall prognosis for CRC patients remains poor [2]. Therefore, there is an urgent need to develop novel therapeutic approaches for CRC. To achieve this, a deeper understanding of the molecular and genetic networks that control the initiation and progression of CRC is imperative.

ZNF217 gene is an oncogene newly cloned in the 20^th^. It locates in the chromosome 20q13.2 and codes a Kruppel-like transcription factor of zinc finger protein family [3]. ZNF217 protein contains 8 predicted Kruppel-like C2H2 zinc finger motifs and a proline-rich region [4]. An increasing number of studies have shown that members of Zinc finger protein family play important roles in the development of a variety of cancers [5]. Many researches have proved that copy number increase of chromosome 20q13.2 is associated with metastasis of CRC [6] and ZNF217 is upregulated in colon cancer as measured by laser capture microdis section and multiplex quantitative real-time PCR [7].

MicroRNAs (miRNAs) are non-coding, 18 to 24 nucleotide long, single-stranded RNAs that have the ability to negatively regulate the expression of genes involved in several cellular processes, including cell proliferation, apoptosis, migration, invasion, and stress response [8, 9, 10, 11, 12]. It has been shown that abnormal patterns of miRNA expression are present in many human carcinomas [13] and associated with the pathogenesis, progression, and natural history of several cancers [11, 14]. Emerging data suggest that miRNAs may function as oncogenes or tumor suppressor genes and play critical roles in cancer development [15]. One study presents evidences that ZNFs are regulated at post-transcriptional level in breast cancer by miR-181a, which directly targets the coding regions of ZNFs [4].

In this study, using bioinformatic algorithms and luciferase reporter assay, we found that ZNF217 is a target of miR-203, a tumor suppressor miRNA. To explore the potential roles of ZNF217 as a novel prognostic biomarker for CRC and its regulation by miR-203 miRNA in CRC tissues and paired normal colorectal tissues, we performed in vitro experiments and confirmed that 1) ZNF217 can promote proliferation, invasion and migration of CRC cell lines and 2) ZNF217 as well as its effects in CRC cell lines are downregulated by miR-203, hoping to further elucidate the mechanism of CRC development and provide novel findings for targeted treatment of CRC.

## Materials and Methods

### Tissue samples

A total of 82 CRC patients who underwent surgical resection of tumors for CRC between July 2004 and March 2009 in the Department of General Surgery, Qilu Hospital of Shandong University, Jinan, China, were recruited for this study. All patients’ data were obtained from clinical and pathologic records, including age, sex, tumor size, differentiation, location, invasion depth and metastasis, as well as tumor-node-metastasis (TNM) stage. The postoperative pathologic staging of each subject was determined according to the 7th edition of the Union for International Cancer Control (UICC) tumor-node-metastasis (TNM) staging system for CRC. The resected tumor tissues and paired adjacent non-cancerous tissues (at least 5 cm away from the tumor margin) were immediately collected, frozen in liquid nitrogen and stored at -80°C. No patients received chemotherapy or radiotherapy before the surgery. This study was approved by the Ethics Committee of Qilu Hospital, Shandong University and written informed consents were obtained from all enrolled patients.

### Immunohistochemistry staining and evaluation for ZNF217

Immunohistochemistry (IHC) was used to detect ZNF217 expression in paraffin-embedded CRC tissues. Paraffin-embedded HCC tissues were sliced as 5 μm sections baked at 65°C for 2 h, and deparaffinized using standard procedures. After antigen retrieval and washing with Tris buffer, ZNF217 primary antibody (Biosynthesis Biotechnology CO, LTD, Beijing China) was applied to slides and expression of ZNF217 was reviewed by incubation with a peroxidase-conjugated goat anti-rabbit antibody (Zhongshan Goldenbridge Biotechnology, Beijing, China) following the manufacturer’s guidelines.

ZNF217 staining was assessed under a light microscope by two independent investigators who were unaware of the clinical outcomes. Staining was considered positive for ZNF217 when a strong correlation was evident in the cytoplasm. Tissues were scored semi-quantitatively by counting the positive cytoplasm of 10 separate fields at 400 X magnification in the areas with the highest density of positive cytoplasm. The appropriate cutoff score was obtained using analysis of receiver operating characteristic (ROC) curves plotted by taking the percentage scores of tumor or adjacent non-tumor tissue as independent variables. The score closest to both maximum sensitivity and specificity, [i.e., the point (0.0,1.0) on the curve] was selected as the cut-off score. Samples with staining score above or below the cutoff score was classified as positive or negative, respectively.

### Cell culture and transfection

CRC cell lines (HT-29, SW480, and SW620) and human embryonic kidney (HEK) 293T cell line were purchased from the Type Culture Collection of the Chinese Academy of Sciences (Shanghai, China), and HCT116 cell line was purchased from Shanghai Institute of Biochemistry and Cell Biology (China). All the cell lines were cultured in Dulbecco’s modified Eagle’s medium (DMEM; Hyaline, UT) containing 10% fetal bovine serum (Gibco, Carlsbad, CA) at 37°C in an incubator supplemented with 5% CO_2_.

Transfection was performed with Lipofectamine 2000 reagent (Invitrogen) following the manufacturer’s protocol. A final concentration of 50 nM miRNA, 100 nM (siRNA) and their respective negative controls were used for each transfection.

### Prediction of candidate miRNAs and luciferase reporter assay

The two most widespread and web-based bioinformatic algorithms (TargetScan and micrornaorg) were used to predict candidate miRNAs targeting the nucleotide sequence of the 3’-untranslated region (UTR) of ZNF217 mRNA. To verify their effectiveness, a luciferase reporter assay was carried out using the pmiR-REPORTTM vectors (RiboBio, Guangzhou, China) containing wild type (WT)-ZNF217 3’-UTR sequence or mutant (MUT)- ZNF217 3’-UTR sequence. HEK293T cells were transiently cotransfected with miR-203 mimics/miR-negative control and WT-ZNF217 3’-UTR vector/MUT ZNF217 3’-UTR. Luciferase activities were measured using the Dual-Luciferase assay kit (Promega, Madison, WI) 48 h after transfection according to the manufacturer’s instructions.

### Real-time RT-PCR and Western blot

Total RNA was extracted using TRIzol reagent (Invitrogen, Carlsbad, CA) according to the manufacturer’s protocol. All of the manipulations of the RNA were carried out under RNase-free conditions. RNA concentration was measured using a BioPhotometer plus (Eppendorf, Hamburg, Germany) at 260 nm, and the isolated RNA was stored at -80°C until use. For the analysis of ZNF217 mRNA expression. A total of 1 µg RNA was reverse transcribed into cDNA using the SuperScript kit (Toyobo, Osaka, Japan)and qRT-PCR analyses were performed using SYBR Green (Toyobo, Osaka, Japan) and an ABI PRISM 7500 Sequence Detection System (Applied Biosystems, Foster City, CA) according to the manufacturer’s instructions. ZNF217 mRNA level was normalized to β-actin and the fold changes in ZNF217 mRNA expression were quantified using the 2^-ΔΔCT^ relative quantification method. The primers used for RT-qPCR of ZNF217 were forward,5’-ATGTTACTCCTCCTCCGGATG-3’ and Reverse,5′-ACACTTGGCCTGTATCTCA-3’. All above primers were from BioSune, Shanghai, China.

For miR-203 expression, cDNA was synthesized using gene-specific primers (Ribobio, Guangzhou, China) and the M-MLV RT kit (Invitrogen, Carlsbad, CA, USA) in a 20-μl reaction. The RT reaction reagents contained 1 μg RNA template, 1 μl 10 mM dNTP mix, 2 μl 0.1 M DTT, 4 μl 5× first-strand buffer, and 1 μL 40 U/μl RNase inhibitor. The volume was adjusted with RNA-free H2O. The reverse-transcription reaction was performed in triplicate to remove any outliers. MiR-203 expression was assessed using qRT-PCR and an ABI PRISM 7500 Sequence Detection System The fold changes in miRNA expression were determined using the 2^−ΔΔCT^ method; the expression was normalized to the U6 small nuclear RNA expression level. The primers used for RT-qPCR of miR-203 were miR-203 forward 5’-GTGAAATGTTTAGGACCACTAGAA-3’, U6 forward 5’-CGCTTCGGCAGCACATATAC-3’ and the universal reverse primer 5’-GCGAGCACAGAATTAATACGAC-3’.

Total proteins were extracted from cultured cells using RIPA buffer containing PMSF and quantified using BCA protein assay kit (Beyotime, Haimen, China). A total of 30 μg proteins were subjected to SDS-PAGE and transferred onto PVDF membranes. After blocking, the membrane was incubated with mouse anti-ZNF217 monoclonal antibody (Abcam, Southampton, UK) or mouse anti-β-actin monoclonal antibody (Santa Cruz Biotechnology, Santa Cruz, CA, USA) followed by incubation with HRP-conjugated secondary antibodies (Santa Cruz Biotechnology, Santa Cruz, CA, USA). Signals were determined by a chemiluminescence detection kit (Amersham Pharmacia Biotech, Piscataway, NJ).

### Cell proliferation assay

Cell proliferation was measured with a methyl-thiazolyltetrazolium (MTT) assay. Twenty-four hours after transfection, cells were seeded at a density of 5×10^3^/well into 96-well plates. After cultured for 24, 48, 72, 96 and 120 h, cells were incubated with 20 µL MTT (5 mg/mL) for 4 h at 37°C. The formed crystals in the cells were volatilized by incubating with 150 µL dimethyl sulfoxide for 10 min at room temperature and quantified by measuring the optical density at 490 nm using an enzyme-linked immunosorbent assay reader (Tecan, Switzerland).

### Cell invasion and migration assay

The invasive and migratory potentials of the cells were evaluated using transwell inserts with pores of 8 μm (Corning). For invasion assay, 24 h after transfection, 3.0 × 10^5^ cells in serum-free medium were added to the upper insert pre-coated with matrigel matrix. 500 μL 10% FBS medium was added to the lower chamber. After incubation for 48 h, non-invading cells were removed from the upper surface of the transwell membrane with a cotton swab, and the invaded cells on the lower membrane surface were fixed in methanol, stained with 0.1% crystal violet, photographed, and counted. Cell migration assay was performed using similar procedures except that 2 × 10^5^ cells were added into non-coated inserts. Cells in six random fields at 200 X magnification for each insert were counted. The assays were conducted in triplicate.

### Statistical analyses

The Student’s t test was used to analyze the differences in ZNF217 expression between the tumor and normal tissues. Correlations between ZNF217 expression and clinicopathological features were analyzed by a nonparametric test: Mann–Whitney U test between two groups and Kruskal–Wallis test for three or more groups. The χ2 and Fisher’s exact tests were performed to determine the associations between ZNF217 expression and clinicopathological parameters. Overall survival curve was calculated by the Kaplan-Meier method and the survival differences of patient subgroups were compared by the log-rank test. Cox regression multivariate analysis was performed to estimate the independent prognostic factors for survival prediction. The correlation between ZNF217 and miR-203 was determined by Pearson’s correlation analysis. Statistical analyses and graphing were conducted using SPSS version 17.0, Microsoft excel and GraphPad Prism software. P < 0.05 was considered as significant difference.

## Results

### ZNF217 expression is correlated with clinicopathological features of CRC

IHC analysis of 82 cases of CRC and their corresponding noncancerous tissues showed that positive staining for ZNF217 was seen in the cytoplasma of CRC cells and corresponding non-cancerous mucosa cells (Fig. 1A). The mean percentages of cells stained positive for ZNF217 in cancerous and corresponding non-cancerous mucosa were 76.3% and 38.9%, respectively. By comparing the percentage of positive cells, it was determined that ZNF217 expression in colorectal carcinoma was statistically higher than that in the adjacent non-cancerous mucosa (P < 0.001; Fig. 1B).

**Figure 1:** IHC staining of ZNF217 in CRC. (A-Left) Cytoplasma staining of ZNF217 in CRC cells. (A-Right) Lack of ZNF217 expression in normal colonic epithelial cells. (B) The percentage of positively stained cells in cancer and adjacent normal tissues (*P < 0.05, **< 0.01). (C) Kaplan–Meier analysis of overall survival in CRC patients according to ZNF217 expression level. The ZNF217 positive group (n = 55) showed significantly shorter survival compared with the negative group (n = 27; P = 0.0405: log-rank test).

Correlation analysis revealed that ZNF217 expression was positively correlated with tumor size, depth of invasion, and lymph node, (P < 0.05), but not with patient age, gender, histology grade, and distant metastases (P > 0.05; Table 1). Furthermore, Kaplan–Meier test showed that patients with positive ZNF217 staining had shorter survival than those with negative ZNF217 staining (P = 0.028; Fig. 1C).

**Table 1:** Association between patients, characteristics and ZNF217 expression in 82 CRC cases.

**Clinicopathologic variable**	**ZNF217 expression**		**Total**	**χ^2^**	**P**
** **	**Positive(n = 55)**	**Negative(n = 27)**		** **	** **
Age(years)					
≥55	42	19	61	0.406	0.524
<55	16	5	21		
Gender					
Male	26	14	40	1.239	0.266
Female	32	10	42		
Tumor size(cm)					
≥5	21	15	36	3.784	0.042
<5	36	10	46		
Histology grade					
Well and moderate	38	21	59	1.467	0.226
Poor	18	5	23		
Depth of invasion					
Muscle	8	10	18	4.701	0.03
Whole wall	46	18	64		
Positive lymph nodes					
Yes	31	8	39	6.148	0.01
No	23	20	43		
Metastasis to other organs					
Present	18	6	24	0.965	0.326
Absent	37	21	58		
Duke, staging					
A+B	28	17	45	3.488	0.062
C+D	30	7	37		

Well and moderate:well and moderately differentiated; poor: poorly differentiated

### Reduction of ZNF217 expression represses CRC cell proliferation, migration and invasion

To measure the biological properties of ZNF217 in CRC cells, we tested proliferation and motility of CRC cells under the condition of siRNA mediated knockdown of ZNF217 gene. First, we examined the expression level of ZNF217 in a panel of CRC cell lines, including HCT-116, HT-29, SW620 and SW480. The results showed that ZNF217 expression level was the highest in SW480 cells and the lowest in HT29 cells among all tested cell lines (Fig. 2A). Based on this expression pattern, we therefore chosed SW480 for further studies. We transiently modulated ZNF217 expression by transfecting siRNA in SW480 cells and found that siRNA-mediated ZNF217 silencing decreased cell proliferation (Fig. 2B) and impaired cell migration and invasion abilities (Fig. 2C). Taken together, our observations indicated that ZNF217 could promote proliferation, migration and invasion of CRC cells.

**Figure 2:** Effects of ZNF217 on proliferation, migration and invasion of SW480 cell lines (A) Expression of ZNF217 in CRC cell lines. (B) Reduction of ZNF217 expression by transfecting siRNA-ZNF217 significantly inhibited proliferation (* P < 0.05) and (C) migration and invasion of SW480 cells (200× magnification, * P < 0.05) in comparison with parental and negative controls.

### ZNF217 were directly targeted by miR-203

Using online miRNA target prediction databases (microrna.org and Targetscan), we found that ZNF217 was a potential target of miR-203 (Fig. 3A). To verify this finding, we constructed luciferase reporters of WT and Mut 3’-UTR of ZNF217 and performed luciferase activity assay in HEK293T cells. The results showed that transfection of miR-203 mimics significantly inhibited the expression of WT but not Mut 3’-UTR of ZNF217 in HEK293T cells (Fig. 3B). Consistent with these results, transfection of miR-203 mimics diminished the endogenous expression of ZNF217 at both mRNA and protein levels in SW480 cells (Fig. 3C and 3D). Moreover, in the analyzed panel of 30 CRC patients, we observed an inverse correlation between ZNF217 and miR-203 expression in CRC tissues and their adjacent normal tissues (Fig. 4E, r = 0.792, P < 0.01; Fig. 3E). Taken together, these data strongly suggested that miR-203 negatively regulates ZNF217 expression via directly targeting its 3’-UTR sequence.

**Figure 3:** MiR-203 negatively regulates ZNF217 expression via the ZNF217 3’-UTR. (A) The putative miR-203 binding sequences in ZNF217 3’-UTR. (B) Luciferase activity assay was performed for the HEK293T cells cotransfected with pmiR-REPORTTM vectors containing WT-ZNF217 3’-UTR or MUT-ZNF217 3’-UTR sequences and miR-203 mimics. Data are presented as normalized fold change in luciferase activity. (C, D) ZNF217 mRNA and protein were determined in SW480 cells transfected with miR-203 mimics or miR-negative control by qRT-PCR and Western blot, respectively. (E) Inverse correlation between ZNF217 mRNA expression and miR-203 levels in CRC tissues was analyzed using Pearson’s correlation analysis.

**Figure 4:** Effects of miR-203 on proliferation, migration and invasion of SW480 cell lines. (A) Ectopic expression of miR-203 by transfecting miR-203 mimics significantly reduced proliferation of SW480 cells, in comparison with parental and negative controls (* P < 0.05). (C) Ectopic expression of miR-203 notably inhibited cell migration and invasion of SW480 cells (200×magnification, * P < 0.05). Inversely, inhibition of miR-203 expression by transfecting miR-203 inhibitors simultaneously (B) promoted proliferation (*P < 0.05) and (D) migration and invasion of SW480 cells, compared with parental and negative controls (200×magnification, *P < 0.05). Figure is a representative of 3 experiments with similar results.

### Effect of miR-203 on CRC cell proliferation, migration and invasion

To validate whether miR-203 could regulate CRC cell proliferation, we performed a proliferation assay in SW480 cells transfected with miR-203 mimics or its negative control, and found that increased expression of miR-203 significantly inhibited proliferation, (Fig. 4A), motility (Fig. 4B), as well as invasion of SW480 cells. Inversely, downregulation of miR-203 in inhibitors-transfected SW480 cells apparently promoted proliferation, motility and invasion of SW480 cells (Fig. 4C).

### Overexpression of miR-203 partially reinforces ZNF217-induced proliferation, migration and invasion of CRC cells

To further explore ZNF217 mediated-tumorigenic effects are regulated by miR-203, we co-transfected SW480 cells with ZNF217 siRNA in combination with miR-203 mimics. We observed synergistic inhibitory effects on ZNF217 expression (Fig. 5A), as well as proliferation, (Fig. 5B), migration and invasion (Fig. 5C) of SW480 cells co-transfected with ZNF217 siRNA and miR-203 mimics in comparison with SW480 cells transfected with either ZNF217 siRNA or miR-203 mimics alone. Taken together, these results indicated that functions of ZNF217 as a potent oncogene are regulated by miR-203.

**Figure 5:** Functional effects of ZNF217 downregulation and miR-203 upregulation on SW480 cells. (A) Effective suppression of ZNF217 protein expression by ZNF217 siRNA and miR-203 mimics respectively and combinedly. Note that ZNF217 expression is more efficiently suppressed by combined treatment. Suppression of ZNF217 simultaneously resulted in (B) significant inhibition of cell growth and (C) migration and invasion (200×magnification) of SW480 cells compared with negative controls. Note the synergistic inhibitory effect of combination of ZNF217 siRNA and miR-203 mimics, compared with either of them alone (*P < 0.05).

## Discussion

ZNF217 is a recently identified member of zinc finger protein family. It mainly functions as a transcriptional regulatory factor involving in the regulation of tumor occurrence and development [16]. ZNF217 possesses several diverse structural domains including eight C2H2 zinc finger DNA-binding motifs as well as a proline-rich (16–20%) domain located at residues 757–1,005. Prolinerich domains have been shown to function as transcriptional activators in many genes such as CTF/NF-1 [3]. ZNF217 gene has been extensively studied in breast cancer [4, 17], ovarian cancer [18, 19, 20], esophageal squamous cell carcinoma [21], gastric cancer [22, 23, 24] and prostate cancer [25, 26], but not in CRC. In Addition, increased copy number of chromosome 20q13.2 has been found to be associated with metastasis of CRC. Thus, it is especially worthwhile to explore its potential roles in CRC development.

In the present study, we found that ZNF217 expression at both mRNA and protein levels was significantly higher in colorectal tumor tissues than in its matched non-tumor tissues and its overexpression was associated with malignant clinicopathological features and short survival of CRC patients, indicating that ZNF217 functions as an oncogene in CRC.

Most cancer patients are died of complications arising from metastasis. Therefore, targeting metastatic diseases is a pivotal anti-cancer strategy. Many studies have revealed that zinc finger proteins that play critical roles in the processes of tumor invasion and metastasis including ZNF217 can be regulated by a variety of genes [27, 28]. In the present study, we found that knockdown of ZNF217 by siRNA led to reduced proliferation, invasion and migration of CRC cells in vitro. These results reveal the oncogenic features of ZNF217 in CRC. Indeed, it has been reported that tumor cells HO-8910, LNCaP, and DU145 [26] as well as breast cancer tissues [4] constructively express high level of ZNF217. Krig et al reported that mis-regulation of E-cadherin and as yet uncharacterized ZNF217 target genes [29] could account for the alterations in cellular immortalization, apoptosis resistance, resistance to chemotherapeutic agents, and Akt phosphorylation in cells with high expression level of ZNF217. Although hundreds of genes are potential targets of ZNF217 and consensus binding sites have been proposed, the specific genes regulating ZNF217 expression are little known.

Accumulating evidences indicate that the aberrant expression of miRNAs is linked to the development of CRC [30, 31, 32]. Sophisticated computer-based approaches for miRNA identification and target prediction as well as validation techniques to confirm these predictions have contributed greatly to the discovery of new miRNAs and their functional characterization. Consequently, small molecule mediated dysregulation of miRNA emerges as a potential new therapeutic approach for human diseases including cancer [33]. Among human cancer-related miRNAs, miR-203 has attracted significant attention because it is expressed aberrantly in a variety of cancers. In our study, we identified for that miR-203 was markedly down-regulated in human CRC and restoration of miR-203 expression could inhibit proliferation, invasion and migration of SW480 cells. On the contrary, transfection of miR-203 inhibitor stimulated proliferation, invasion and migration of SW480 cells. These findings suggest that miR-203 is involved in the metastasis processes of CRC and are in agreement with the previous studies showing that miR-203 were expressed at lower than normal level in some cancers [34, 35, 36, 37]. However, miR-203 have been reported to exert a oncogene function in kidney and bladder cancers [38] and pancreatic adenocarcinoma [39]. The discrepancies in miR-203 functions in different types of cancer may reflect the differences of cellular context or alternatively targeted genes.

The current study provides several lines of evidences that ZNF217 is a novel target of miR-203 and their antagonistic interaction plays an important role in the development of CRC. First, the luciferase reporter assay demonstrated that luciferase activity under the control of the ZNF217 3’UTR could be regulated by miR-203. Secondly, an inverse correlation between ZNF217 and miR-203 levels was observed in CRC tissues. Thirdly, overexpression of miR-203 suppressed ZNF217 levels and led to reduced cell proliferation, migration and invasion in CRC cell lines.

In summary, in this study we demonstrated that ZNF217 is frequently upregulated in CRC and a potential oncogene for CRC development. Meanwhile, our research described ZNF217/miR-203 link and provided a potential mechanism for ZNF217 dysregulation and contribution to CRC cell invasion. These findings open up the possibility of applying miR-203 toward clinical CRC treatments.
